# Detection of *mecA* and 16S rRNA Genes Using Real-Time PCR Can Be Useful in Diagnosing Iliopsoas Abscess, Especially in Culture-Negative Cases: RT-PCR for Iliopsoas Abscess

**DOI:** 10.1155/2022/2209609

**Published:** 2022-02-11

**Authors:** Hyonmin Choe, Naomi Kobayashi, Yohei Ito, Hiroyuki Ike, Taro Tezuka, Masanobu Takeyama, Yusuke Kawabata, Yutaka Inaba

**Affiliations:** ^1^Yokohama City University Department of Orthopaedic Surgery, 236-0004 3-9 Fukuura, Kanazawa-ku, Yokohama City, Kanagawa, Japan; ^2^Yokohama City University Medical Centre Department of Orthopaedic Surgery, 232-0024 4-57 Urahune-cho, Minami-ku, Yokohama City, Kanagawa, Japan

## Abstract

The rapid detection of etiological agents is important for the successful treatment of iliopsoas abscess (IPA). The purpose of this study was to investigate the clinical utility of a real-time polymerase chain reaction (PCR) that targets the *mecA* gene for methicillin-resistant staphylococci (MRS) and the 16S rRNA gene for pan-bacteria. Our retrospective diagnostic study included 22 patients exhibiting IPAs and four patients with noninfectious iliopsoas mass regions who underwent computerized tomography or ultrasonography-guided biopsy and/or surgical treatment. Clinical symptoms, serum data, imaging analysis, and tissue microbiological culture were utilized for the diagnosis of IPA. The diagnostic accuracy of real-time PCR was determined based on the diagnosis of IPA and microbiological culture results. The microbiological culture was positive for 12 IPA cases that included 2 MRSA infections. Among 12 culture-positive IPA cases, 16S rRNA-PCR was positive in 12 and MRS-PCR in two. Among 10 culture-negative IPA cases, including 3 TB cases, 16S rRNA-PCR was positive in 8 and MRS-PCR in 2. In noninfectious iliopsoas mass patients, neither 16S rRNA nor MRS-PCR detected bacterial DNA. The sensitivity, specificity, positive predictive, and negative predictive values of 16S rRNA-PCR for diagnosing IPA were 0.91, 1.00, 1.00, and 0.67, respectively, while those for the diagnosis of MRS infection with MRS-PCR were 1.00, 0.92, 1.00, and 0.50, respectively. Real-time PCR targeting bacterial DNA can detect bacterial DNA in culture-negative cases and offer improved detectability of MRS infection in IPA patients.

## 1. Introduction

Iliopsoas abscess is a relatively rare disorder that requires emergent diagnosis and extensive antibiotic treatment. The determination of causative pathogens is essential for the successful treatment of iliopsoas abscess. *Staphylococcus aureus* and *Escherichia coli* (*E. coli*) are 2 major causative organisms, but any kind of bacterial species can cause iliopsoas abscess. Bacterial culture reportedly shows false-negative results in 25% of patients, which can be attributed to the viable but nonculturable (VBNC) condition of causative bacteria due to prophylactic use of antibiotics and biofilm formation [1]. Although the clinical utility of real-time polymerase chain reaction (PCR) targeting *Mycobacterium tuberculosis* (TB) has been widely documented, diagnosis of other bacteria is still based on microbiological culture, making it difficult to identify the causative organism and rapid and adequate antibiotic treatment [1, 2].

Methicillin resistance has been increasing over the last two decades [3–5]. If the microbiological culture shows false-negative results, methicillin-resistant staphylococcus- (MRS-) targeting antibiotics must be considered in all iliopsoas abscesses to cover the most likely causative bacteria. Since real-time PCR has been reported as a useful tool for the diagnosis of infections with VBNC [6, 7], real-time PCR can improve the diagnostic accuracy of iliopsoas abscess and antibiotic selection. In addition, since real-time PCR detects both live and dead bacterial DNA [8, 9], it can detect bacterial DNA in patients with prior initiation of antibiotic treatment.

All bacteria possess 16S rRNA, a pan-bacterial DNA [10, 11]. Targeting the 16S rRNA gene makes it possible to specifically identify bacterial infections using real-time PCR [10–12]. In addition, by identifying the *mecA* that is specific for the methicillin-resistant bacteria, it is possible to specifically identify the presence of MRS and apply it to the selection of antibacterial agents [13–15]. Another advantage of real-time PCR is that it can be conducted within few hours after sampling [13, 16]. While the advantages of high accuracy and rapidity of real-time PCR have been sufficiently proven in the diagnosis of tuberculosis (TB) [17], they have been less demonstrated in other bacterial infections, especially in IPA.

We hypothesized that real-time PCR-based genetic diagnosis can contribute to the accurate diagnosis of culture-negative IPA. Therefore, the purpose of the current study was to investigate the utility of the 16S rRNA real-time PCR for the diagnosis of IPA and that of *mecA* gene real-time PCR for the complementary detection of MRS infection.

## 2. Participants and Methods

This retrospective study was approved by our institutional review board (B210500004). From July 2009 to December 2020, 32 patients (16 females/16 males; mean age: 67.8 years (range: 44–86)) in whom a iliopsoas mass region was detected via computed tomography (CT) and/or magnetic resonance imaging (MRI) in our hospital—who were thereby suspected of having an iliopsoas abscess—were selected for this retrospective study. Among 32 patients, 6 were excluded because surgical specimen or fluid was not submitted for the assessment of real-time PCR in these 6 patients (Figure 1).

In our attempt to diagnose IPA, the clinical symptoms of iliopsoas pain, unknown fever, improvement of symptoms after antibiotic treatment, serum data of white blood cell (WBC) count (cells/mm^3^), serum C-reactive protein (CRP) values (mg/dl), albumin level (g/dl), imaging analysis, microbiological culture for sampling abscess, microbiological culture, and histopathological assessment for surgical specimens were investigated. Definitive diagnosis of IPA was based on the serum CRP level, MRI findings associated with spinal discitis, microbiological and histopathological results for abscess or tissue, and exclusion of benign or malignant tumors. Of the 26 patients of the study cohort, 22 received a definitive diagnosis. Four patients were diagnosed as having a noninfectious iliopsoas mass region, of which two were idiopathic iliopsoas hematomas, one iliopsoas bursitis, and one malignant lymphoma (Figure 1).

The total cohort consisted of 13 female and 13 male subjects with a mean age of 67 years (range: 44–86 years) who underwent computerized tomography- (CT-) or ultrasonography- (US-) guided biopsy and/or surgical treatment. Mean WBC count, CRP, and albumin level were 10310 (cells/mm^3^), 9.8 (mg/dl), and 3.1 (g/dl), respectively. All sampled abscesses were submitted for microbiological culture, histopathological assessment for neutrophil infiltration (not applicable in 8 cases), and real-time PCR.

### 2.1. Microbiological Culture

All specimens were cultured using standard microbiological aerobic and anaerobic techniques. The direct plating method was performed alongside simultaneous enrichment using the Gifu Anaerobic Medium semisolid broth culture method for up to five days in a Nissui Tube (Nissui Pharmaceutical, Tokyo, Japan). If samples were not cultured after five days, incubation was extended for up to 14 days. The bacteria were allowed to grow, and the VITEK 2 compact device (Biomerieux, Inc., Durham, NC, USA) was used for automated identification of microorganisms, per the manufacturer's instructions.

### 2.2. Histopathological Examinations

Infiltration of neutrophils or existence of bacteria was regarded as presence of infection.

### 2.3. Real-Time PCR

DNA extractions were performed using a Bio Robot EZ1 DNA® investigator kit with a Bio Robot EZ1® (Qiagen Inc., Valencia, CA) or QIAamp DNA Mini Kit® (Qiagen Inc., Valencia, CA), in accordance with the manufacturer's instructions.

From July 2009 to December 2013, and from January 2016 to December 2020, the LightCycler® system (Roche Diagnostics, Mannheim, Germany) was used to analyze real-time PCR assays. Briefly, MRS-PCR using an MRS aureus detection kit (Roche Diagnostics, Mannheim, Germany) targeting the *mecA* gene and broad-range detection of bacterial DNA was carried out by a set of broad-range forward and reverse PCR primers that targeted a part of the 16S rRNA gene previously described [18, 19]. The following program settings were used for the real-time PCR procedure: an initial hot start at 95°C for 10 minutes, followed by 45 cycles at 95°C for 10 seconds, 55°C for 10 seconds, and 72°C for 12 seconds. The differences between the threshold cycles (Ct) for the negative control (sterile water) and the case samples were calculated as ΔCt. Moreover, ΔCt > 2 cycles was defined as positive in 16S rRNA-PCR [14, 18, 20].

From November 2013 to January 2016, the LightCycler NanoVR system (Roche Diagnostics, Mannheim, Germany) was used to analyze real-time PCR assays. Primer and prove sets of MRS-PCR and 16S rRNA-PCR were utilized as previously described [21]. After an initial hot start incubation at 95°C for 10 min, 40 cycles of PCR amplification were performed with the following parameters: 95°C for 10 s and 60°C for 30 s. DNase- and RNase-free water was used in all cases to avoid contamination.

### 2.4. Data Analysis

The differences in mean WBC count, CRP values, and albumin level between iliopsoas abscesses and noninfectious iliopsoas mass regions were statically analyzed using Student's *t*-test. The accuracy (sensitivity and specificity, positive predictive value (PPV), negative predictive value (NPV), and accuracy) of 16S rRNA-based real-time PCR was assessed by comparing the PCR result with infectious diagnosis of IPA, while the accuracy of the MRS-PCR was investigated by comparing the PCR result with culture results.

## 3. Results

### 3.1. Patient Background and Serum Data

Between IPA patients and noninfectious iliopsoas mass patients, there was no difference in age and gender (Table 1). The comorbidities of IPA patients included pyogenic spondylitis (*n* = 5), spinal instrument infection (*n* = 2), endometrial cancer (*n* = 2), perirenal abscess (*n* = 1), rheumatoid arthritis (*n* = 1), and cirrhosis (*n* = 1). The total protein, WBC, and CRP value were not significantly different between IPA patients and noninfectious iliopsoas mass patients (6.7 vs. 7.0 (*p* = 0.52), 9.0 vs. 13.4 (*p* = 0.36), and 10854 vs. 6950 (*p* = 0.27), respectively); however, the albumin level was significantly lower in IPA patients, compared with noninfectious iliopsoas mass patients (2.9 vs. 3.7, respectively; *p* = 0.04) (Table 1 and Figure 2), which indicates undernutrition in IPA patients.

### 3.2. Microbiological Culture and Real-Time PCR

Microbiological culture was positive for 12 IPA patients. The following cultures were identified: 4 streptococci (2 agalactiae, 1 beta group, and 1 dysgalactiae), 3 MSSA, 2 MRSA, 1 *Staphylococcus warneri*, 1 *Bacteroides vulgatus*, and 1 *Propionibacterium* infections. Among 12 culture-positive IPA patients, 12 exhibited positive 16S rRNA-PCR and two exhibited positive MRS-PCR (Table 2). Among 10 culture-negative IPA patients, including 3 TB patients, 16S rRNA-PCR was positive for eight patients and MRS-PCR was positive for two (Table 2). In four patients with noninfectious iliopsoas mass, neither 16S rRNA- nor MRS-PCR-detected bacterial DNA was found. The sensitivity, specificity, positive and negative predictive values, and accuracy of 16S rRNA-PCR for diagnosing IPA were 0.91, 1.00, 1.00, 0.67, and 0.92, respectively, while those for the diagnosis of MRS infection with MRS-PCR were 1.00, 0.92, 1.00, 0.50, and 0.92, respectively (Table 3).

### 3.3. A Representative Case of Culture-Negative IPA

A 40-year-old woman diagnosed with juvenile idiopathic arthritis at 35 years of age, who complained of right hip pain and was suspected of having an iliopsoas abscess, was referred to our hospital. At presentation, 8 mg of weekly MTX, 5 mg of daily PSL, and tocilizumab every other week were administered for the treatment of JIA with serum CRP of 4.3 mg/ml and albumin of 4.0 g/dl. Due to her past history of septic shock, she had been taking oral antibiotic of trimethoprim-sulfamethoxazole (TS) twice per week for a prophylactic purpose. Past surgical treatment included bilateral total knee and hip arthroplasty for hip arthritis 20 years ago and total hysterectomy and adnexectomy for uterine adenomyosis and ovarian endometriosis 3 years ago. Computed tomography images showed iliopsoas abscess (Figures 3(a) and 3(b)). A fluid sample was obtained by abscess puncture and assessed via microbiological culture and real-time PCR assay. Despite a culture-negative result, bacterial DNA was detected by 16S rRNA-PCR and MRS infection was determined by MRS-PCR (Figures 3(c) and 3(d)). Since abscesses widely expanded in the retroperitoneum and compressed the femoral neurovascular structures (Figures 3(a) and 3(b)), surgical debridement of iliopsoas abscess was performed with an ilioinguinal approach in supine position. A sample of the walls surrounding the abscess was taken for microbiological culture, histological examination, and real-time PCR. While the microbiological culture was negative, the histopathological examination showed extensive infiltration of neutrophils, indicating acute inflammation caused by bacterial infection. At the postoperative investigation for surgical specimens, MRS-PCR was positive again. Anti-MRS treatment was started with intravenous administration of daptomycin in combination with rifampicin plus minocycline. Daptomycin was changed to linezolid after 2 weeks of administration. After 5 weeks of treatment with linezolid, the antibiotics were changed to TS combination after confirming the reduction of CRP value. The mass region of iliopsoas abscess remained for 2 weeks after surgery (Figure 3(e)); however, it had disappeared 3 months after surgery, according to a CT scan (Figure 3(f)). This highlights the importance of appropriate antibiotic selection in IPA treatment, even after surgical treatment.

## 4. Discussion

Iliopsoas abscess is a relatively rare disorder that has a diversity of frequency depending on patients' race, gender, and preexisting diseases [1]. Sequential iliopsoas abscess has been reported in the immunological suppression in rheumatoid arthritis, cervical spondylosis infection, ulcerative colitis, malignant tumor cases, and cardiovascular disorders [22–26]. Our study demonstrated that undernutrition is an indicator for the possible presence of IPA; however, serum inflammatory markers may not be useful to differentiate IPA from other inflammatory responses. These patients require emergent and adequate treatment, including appropriate antibiotic selection [1, 27–30]. Nevertheless, in patients with such immunodeficiency, antibacterial agents are often administered in advance to prevent infectious diseases that may induce a culture-negative condition for IPA, as shown in our representative case of culture-negative MRS IPA.

Preadministration of antibacterial agents also induces false-negative culture results due to the VBNC condition of causative bacteria in infectious diseases [6]. Since the VBNC condition is a state in which the bacteria are different from the general status, amplification by bacterial culture is inhibited, and it becomes difficult to identify the bacteria [6]. By targeting the bacterial gene, real-time PCR is possibly a more accurate means of diagnosis for bacterial infections, compared with microbiological culture, which has limited accuracy in the detection of causative bacteria in IPA patients [1].

It was observed that the iliopsoas abscess was often enlarged, compressing the nerve or blood vessels. Thus, surgical debridement is the most viable option if mass legion exceeds 10 cm in size [1, 29]. However, extensive surgical debridement is difficult while treating iliopsoas abscesses because of the deep anatomical location of the iliopsoas muscle, which is surrounded by the retroperitoneum and blood vessels. Therefore, as shown in the case presentation, long-term administration of effective antibiotics is still a viable strategy for IPA patients after surgical treatment. Thus, sensitive etiological diagnosis is critical in the successful treatment of IPA.

The novelty of this study consists of our assessment of the utility of real-time PCR in the diagnosis and treatment of IPA. Although the utility of real-time PCR has previously been demonstrated, its accuracy for detecting bacterial genes or MRS in IPA patients has not been investigated. The advantages of real-time PCR for detection of bacterial DNA are the rapidity of the procedure and the specificity of detecting the antibiotic resistance gene. IPA in immunocompromised patients may be greatly beneficial in the selection of antibiotics if the presence of MRS can be confirmed within a few hours after tissue sampling. Evidentially, MRS-PCR was positive in two patients who had culture-negative results in our cohort (Table 2). In these cases, the use of antibiotics targeting MRS can be critical in the treatment of IPA (as shown in our case presentation) or for improvement of the mortality rate in patients with severe comorbidities [26]. Furthermore, rapid molecular detection or exclusion of the presence of bacterial DNA may lead to avoidance of unnecessary antibiotics use, which could cause liver dysfunction, renal disorders, and generation of antimicrobial resistance in IPA patients.

Accurate diagnosis is often difficult in orthopedic infections due to their lack of specificity in clinical symptoms or serum examinations [31]. Therefore, synovial fluid testing for the detection of infection-specific immunological proteins or bacterial genes is a widely accepted procedure for improved diagnostic accuracy for orthopedic infections [31–33]. In our IPA patients, except albumin level, the serum test also had only little utility in differentiating IPA from noninfectious iliopsoas mass. Since puncturing the abscess from the infected site is a gold standard for diagnosis of IPA, pan-bacterial 16S rRNA real-time PCR for directly obtained abscesses may contribute to more accurate IPA diagnoses without requiring extra invasion for patients exhibiting iliopsoas mass region.

A limitation of this study is the small number of patients and the study design of retrospective observational research. During the study period, we excluded 6 IPA patients due to lack of assessment in real-time PCR result that may affected the result of our current study. However, our current study firstly demonstrated the accuracy of real-time PCR for the diagnosis of IPA and utility of molecular detection of MRS, although their usage is still limited in research purpose. Another limitation of the study was the fact that the 16S rRNA-PCR required quantitative judgment using Ct values instead of qualitative judgement as in MRS-PCR. This is because we applied DNA polymerase containing a subtle amount of bacterial contamination in the 16S rRNA-PCR procedure, according to the manufacturer's instructions. Nevertheless, in infections such as IPA, where the infection contains a large concentration of bacteria, the difference of the Ct value can be clear, and our procedure may still lead to an accurate diagnosis of IPA. The 16S rRNA region is a region where sequence analysis is greatly advanced; therefore, DNA polymerase without bacterial contamination for the 16S rRNA region, a genetic testing kit for identification of specific bacterial DNA, and/or determination of bacteria according to next-generation sequencing can be expected to contribute to the improvement of diagnosis and treatment of IPA in the near future.

In conclusion, 16S rRNA-PCR can detect bacterial DNA in culture-negative IPA cases, leading to rapid diagnosis of IPA. Therefore, MRS-PCR that targets *mecA* gene can improve detectability and antibiotic selection for MRS infection in IPA patients.

## Figures and Tables

**Figure 1:** Patient enrollment in this study. Among 32 patients with iliopsoas mass region, six were excluded due to lack of real-time PCR results. As a result, 22 patients with iliopsoas abscess and four with noninfectious mass were enrolled in the current study.

**Figure 2:** Serum data in patients with iliopsoas abscess and noninfectious mass. The albumin level was significantly lower in iliopsoas abscess, although there was no difference in total protein, C-reactive protein (CRP), and white blood cell (WBC) count levels. Bars indicate the mean ± standard deviation.

**Figure 3:** X-ray and computed tomography (CT) images at first presentation. Axial image (a) and coronal image (b) of the CT at first presentation show a mass region with a major axis of 10 cm in accordance with the right iliac and psoas muscles that compress the right artery and vein (white arrow). No mass is found around the hip joint. MRS-PCR shows positive for *mecA* gene detection (c) and 16S rRNA gene detection (d) despite a culture-negative result. Intraoperative finding shows the mass region's extensive amount of fluid that compresses the femoral nerve from the retroperitoneum side (e). CT showed residual mass region 2 weeks after surgery (f), which disappeared three months after surgery (g).

**Table 1:** Demographic data.

	Age	Gender	Administration of antibiotic	Comorbidities
Iliopsoas abscess (*N* = 22)	67.5 [12.5]	Female: 11	13	Pyogenic spondylitis: 5 Spinal instrument infection: 2 Endometrial cancer: 2 Perirenal abscess: 1 Rheumatoid arthritis: 1 Cirrhosis:1
Noninfectious iliopsoas mass (*N* = 4)	64.5 [10]	Female: 3	0	Idiopathic iliopsoas hematoma: 2 Iliopsoas bursitis: 1 Malignant lymphoma: 1

**Table 2:** Comparison between methicillin resistant staphylococcus (MRS)-PCR and microbiological culture for detecting MRS infection.

		Microbiological culture			Total
		Positive (*N* = 12)		Negative (*N* = 14)	
		MRS	Bacteria other than MRS		
MRS-PCR	Positive	2	0	2	4
	Negative	0	10	12	22

**Table 3:** Accuracy of real-time PCR for diagnosis of iliopsoas abscess and detection of MRS infection.

	Sensitivity	Specificity	PPV	NPV	Accuracy
16S rRNA-PCR	0.91	1.00	1.00	0.67	0.92
MRS-PCR	1.00	0.92	1.00	0.50	0.92

NPV: negative predictive value; PCR: polymerase chain reaction; PPV: positive predictive value.

## Data Availability

The clinical data used to support the findings of this study are available from the corresponding author upon request.
